The article "Effect of Electroacupuncture Combined with Guizhi Gegen Decoction on Cervical Vertigo and Its Influence on TCD of Vertebrobasilar Artery, Blood Rheology Indexes, and Quality of Life" was retracted in 2023. Reasons: signs of a paper mill; compromised peer review; unreliable results or conclusions.

# Effect of Electroacupuncture Combined with Guizhi Gegen Decoction on Cervical Vertigo and Its Influence on TCD of Vertebrobasilar Artery, Blood Rheology Indexes, and Quality of Life

**DOI:** 10.1155/2021/2676485

**Published:** 2021-09-14

**Authors:** Bo Li, Li Chen, Dongqiang Wang

**Affiliations:** Combined Chinese and Western Medicine Division, Tianjin First Central Hospital, Tianjin 300192, China

## Abstract

Cervical vertigo is a common clinical disease. In this study, we investigated the clinical efficacy of adding the treatment protocol of Gui Zhi Ge Gen Tang and electroacupuncture to the Western medical treatment in cervical vertigo. The results showed that the total effective rate of the study group was higher than that of the control group (*P* < 0.05). After treatment, the vertigo, headache, neck and shoulder pain, daily life and work, and psychological and social adjustment scores were higher in the study group than in the control group (*P* < 0.05). LVA, RVA, and VB were higher in the study group than in the control group after treatment (*P* < 0.05). The whole blood viscosity high cut, whole blood viscosity low cut, and plasma viscosity levels were lower in the study group than in the control group after treatment (*P* < 0.05). After treatment, PF, RF, RE, BP, GH, VT, SF, MH, and HT were higher in the study group than those before treatment (*P* < 0.05). The incidence of adverse reactions was not statistically significant in the study group compared with the control group (*P* > 0.05). This means that electroacupuncture combined with Gui Zhi Ge Gen Tang can effectively increase the blood flow velocity of the vertebrobasilar artery in patients with cervical vertigo and improve their blood rheology and quality of life with definite efficacy and high safety.

## 1. Introduction

Cervical vertigo is a disorder of blood flow and vasospasm triggered by the compression of the vertebral arteries by soft tissue lesions in the cervical spine and neck, sympathetic nerves [1]. The clinical symptoms are mainly paroxysmal vertigo, which can be accompanied by nausea, tinnitus, nystagmus, paresthesia, etc [2]. Cervical vertigo is an important disease affecting the quality of life of modern people, and it is also one of the inducements of cardiovascular diseases such as hypertension and atherosclerosis [3]. At present, the incidence of cervical vertigo is increasing year by year, and the age of onset also tends to be younger. The search for effective treatment options becomes the clinical consensus.

Cervical vertigo falls into the category of “vertigo” in traditional Chinese medicine (TCM). Due to the holistic nature of TCM's dialectical treatment, it has become a featured method for the treatment of cervical vertigo [4]. Guizhi Gegen decoction that comes out of “Treatise on Febrile Diseases” has the effect of releasing muscle. Acupuncture is a characteristic of external treatment in TCM [5]. Modern pharmacology research has shown that acupuncture at acupoints such as Fengchi (GB 20), Dazhui (GV 14), and Baihui (GV 20) can effectively alleviate the hypertonia in the cervical muscle and improve the local blood circulation, thereby effectively relieving the symptoms such as neck discomfort [6]. Due to the complexity of the pathogenesis of cervical vertigo and its clinical characteristics of repeated attacks, a single treatment has its limitations, and now, comprehensive treatment is mainly used in clinical practice. This study combined electroacupuncture and decoction for the treatment of cervical vertigo and the impact on vertebrobasilar artery TCD, blood rheology indexes, and quality of life, which are reported as follows.

## 2. Materials and Methods

### 2.1. General Data

120 patients with cervical vertigo treated in our hospital from October 2019 to October 2020 were selected as the research object, and their clinical data were analyzed retrospectively. According to the difference in treatment methods, they were divided into a study group and a control group. There were 63 patients in the study group, including 34 males and 29 females, with an age of (54.19 ± 13.26) years and a course of (5.42 ± 2.13) years. Also, there were 57 patients in the control group, including 32 males and 25 females, with an age of (54.23 ± 13.52) years and a course of (5.39 ± 2.16) years. There was no statistical significance in the general data between the two groups (*P* > 0.05). All patients signed informed consent forms, and this study has been approved by the Medical Ethics Committee of our hospital.

### 2.2. Inclusion Criteria

(i) Western medicine met the diagnostic criteria of cervical vertigo established in Practical Psychiatry [7]. TCM met the dialectical criteria of cervical spondylosis of vertebral artery type in Guiding Principles for Clinical Research on New Drugs of Traditional Chinese Medicine (for Trial Implementation) [8]. (ii) Age 25∼70 years.

### 2.3. Exclusion Criteria

(i) Patients with severe hypertension and hypotension. (ii) Noncervical vertigo diseases, such as brain-derived, ear-derived, eye-derived, and drug-derived vertigo. (iii) Patients with combined inner ear, vestibular nerve, brain stem, cerebellum, and cerebral lesions. (iv) Pregnancy, lactation, and allergic constitution and other patients who cannot tolerate electroacupuncture treatment. (v) Patients with coagulation disorders.

### 2.4. Treatment Methods

All patients received conventional Western medicine treatment, adding 20 mL Of Shuxuening (Beijing China Resources High-tech Natural Medicine Co., LTD., National drug approval Z11021351) into 250 ml 5% glucose injection, once a day. At the same time, blood pressure and blood glucose were actively controlled.

On the basis of routine treatment of Western medicine, patients in the control group were treated with Guizhi Gegen decoction. The medicinal composition comprises Radix Puerariae 30 g, Radix Cyathulae 30 g, Caulis Spatholobi 30 g, Ramulus Cinnamomi 10 g, Radix Gentianae Macrophyllae 10 g, Radix Paeoniae Alba 10 g, Radix Clematidis 10 g, and Radix Glycyrrhizae Preparata 6 g. The drug was orally taken in the morning and evening twice, 1 dose per day, by decocting with water to 500 ml.

Based on the treatment plan of the control group, patients in the study group were given electroacupuncture (EA) treatment. With the assistance of X-ray, the position of Jiaji points in neck 4∼7 was obtained, and Tianzhu (ST 25), bilateral Fengchi (GB 20), Houxi (ST 34), and Lieque (GB 34) were selected as auxiliary points. The patient took a sitting position and underwent routine disinfection, and Hua Tuo brand 0.30 mm × (25∼40) mm disposable sterile acupuncture needles (produced by Suzhou Medical Products Factory Co., LTD.) were used for acupuncture. The acupoints of Fengchi (GB 30) were perpendicularly inserted into Tianzhu (ST 25) for 30 mm in the direction of the contralateral eyeball and those of Jiaji (EX-B2) of the neck 4–7 for 13 mm in the direction of the spinal column, 5 mm in the direction of Lieque (GB 24) for the finger, and 26 mm in Houxi (GB 34). After getting Qi, the Fengchi (GB 30), Tianzhu (ST 25), and 2 pairs of cervical Jiaji points were selected. The g9805-c low-frequency electronic pulse therapeutic instrument was connected, and the intensity is based on the patient's tolerance, 30 min/time, 1 time/d.

All the patients took 7 d as a course of treatment, and the next course of treatment began after an interval of 1 d. The two groups received continuous treatment for two courses, and then, the clinical efficacy was evaluated.

### 2.5. Observation Indicators

#### 2.5.1. Clinical Efficacy

The criteria for the evaluation of efficacy refer to the Guiding Principles for Clinical Research of New Chinese Medicine (Trial) [8]. i) Recovery: The clinical symptoms and signs such as vertigo were completely disappeared, and the vertebral-basilar artery blood flow velocity test results were restored to normal. Also, the neck movement was unobstructed. ii) Markedly effective: Clinical symptoms and signs such as vertigo disappeared basically, and the vertebral-basilar artery blood flow velocity test results returned to normal. Besides, there was slight discomfort after the neck moved. iii) Effective: The symptoms such as vertigo and vertebral-basilar artery blood flow velocity were improved compared with those before treatment, and the neck movement was obviously impaired. iv) No effect: Compared with those before treatment, the clinical symptoms, vertebral-basilar artery blood flow velocity, and various test indexes were not significantly changed or even worsened.

#### 2.5.2. Evaluation of Symptoms and Functions of Cervical Vertigo Scale (ESCV) Score

Before and after treatment, patients' vertigo, headache, neck and shoulder pain, daily life and work, and psychological and social adjustment were scored according to ESCV [9], and each item was scored according to 5 grades, with a full score of 3 points. The lower the score, the more severe the condition.

#### 2.5.3. Transcranial Doppler Ultrasound (TCD) of the Vertebrobasilar Artery

The TCD of the vertebrobasilar artery was examined in both groups before and after treatment, and the changes of systolic maximum flow velocity (PS) and time-averaged flow velocity (TAMn) of the left vertebral artery (LVA), right vertebral artery (RVA), and vertebral-basilar artery (VB) of patients were observed.

#### 2.5.4. Blood Rheology Indexes

5 mL of fasting venous blood was collected from two groups of patients before and after treatment, and the levels of whole blood viscosity high cut, whole blood viscosity low cut, and plasma viscosity were detected by using the MEN-C200 automatic blood rheology dynamic analyzer.

#### 2.5.5. Quality of Life

Before and after treatment, the MOS item short from health survey (SF-36) [10] was used to assess patients' physical functioning (PF), physical function (role-physical, RF), emotional function (role-emotional (RE), bodily pain (BP), general health (GH), vitality (VT), social functioning (SF), mental health (MH), and health transition (HT). The total score ranges from 0 to 100, and the higher the final score, the better the quality of life of the subjects.

#### 2.5.6. Adverse Effects

The occurrence of adverse reactions during and after treatment in the two groups was compared.

### 2.6. Statistical Methods

All data were processed with SPSS 22.0 statistical software, and GraghPad prism 8 was used to make statistical graphs. Measurement data are expressed as mean ± standard deviation $\left(\bar{x}\pm s\right)$, the independent sample *t*-test is used for comparison between groups, count data are expressed as [*n* (%)], and the chi-square (*χ*^2^) test is performed. The difference is statistically significant when *P* < 0.05.

## 3. Results

### 3.1. Comparison of Clinical Efficacy between the Two Groups

The total effective rate of the study group was 95.24%, and the total effective rate of the control group was 84.21%. The total effective rate of the study group was higher than that of the control group, and the difference was statistically significant (*P* < 0.05, Table 1).

### 3.2. Comparison of ESCV Scores before and after Treatment between the Two Groups

The comparison of vertigo, headache, neck and shoulder pain, daily life and work, and psychological and social adjustment scores before treatment was not statistically significant between the two groups (*P* > 0.05).

After treatment, the scores of vertigo, headache, neck and shoulder pain, daily life and work, and psychological and social adjustment in both groups were higher than those before treatment (*P* < 0.05). Also, the scores of vertigo, headache, neck and shoulder pain, daily life and work, and psychological and social adjustment were higher in the study group than in the control group, and the differences were statistically significant (*P* < 0.05, Table 2).

### 3.3. Comparison of TCD before and after Treatment between the Two Groups

The comparison of LVA, RVA, and VB before treatment was not statistically significant between the two groups (*P* > 0.05). After treatment, LVA, RVA, and VB in both groups were higher than those before treatment (*P* < 0.05). Also, the LVA, RVA, and VB in the study group were higher than those in the control group, with statistical significance (*P* < 0.05, Table 3).

### 3.4. Comparison of Blood Rheological Index Levels before and after Treatment between the Two Groups

The comparison of whole blood viscosity high cut, whole blood viscosity low cut, and plasma viscosity levels before treatment in both groups was not statistically significant (*P* > 0.05). After treatment, the levels of whole blood viscosity high cut, whole blood viscosity low cut, and plasma viscosity in both groups were lower than those before treatment (*P* < 0.05). The whole blood viscosity high cut, whole blood viscosity low cut, and plasma viscosity levels in the study group were lower than those in the control group, and the difference was statistically significant (*P* < 0.05, Table 4).

### 3.5. Comparison of the Quality of Life between the Two Groups before and after Treatment

The comparison of PF, RF, RE, BP, GH, VT, SF, MH, and HT between the two groups before treatment was not statistically significant (*P* > 0.05). After treatment, PF, RF, RE, BP, GH, VT, SF, MH, and HT were higher in the study group than before treatment (*P* < 0.05); however, there was no statistically significant comparison between PF, RF, RE, BP, GH, VT, SF, MH, and HT in the control group after treatment and before treatment (*P* > 0.05, Table 5).

### 3.6. Occurrence of Adverse Reactions in the Two Groups

In the study group, there was 1 case of acupuncture fainting, while in the control group, there was no adverse reaction during the treatment. There were no significant changes in blood and urine routine and liver and kidney function tests in the two groups after treatment. The incidence of adverse reactions in the study group was not statistically significant compared with that in the control group (*P* > 0.05).

## 4. Discussion

The pathophysiology and pathogenesis of cervical vertigo are very complex. At present, there are six main theories, including proprioceptor disorder, sympathetic nerve function stimulation, insufficient blood supply to the basilar artery, migraine related, cervical instability, and humoral factors [11, 12]. Western medical treatment mainly uses vasodilator drugs and sedative drugs. Shuxinin is a medicine with *Ginkgo biloba* extract as the main ingredient, which is mainly used clinically for vertigo, headache, deafness, tinnitus, and amnesia caused by brain marrow disorders. Clinical practice has found that the application of ShuXinNing can improve the clinical symptoms of cervical vertigo to a certain extent, but could not cure fundamentally [13]. With the development of modern TCM, the treatment of cervical vertigo by TCM has achieved remarkable effect in recent years.

Cervical vertigo belongs to the category of “paralysis.” On the one hand, most patients with cervical vertigo are deficient, including deficiency of liver and kidney yin, deficiency of qi and blood, and deficiency of kidney essence [14]. On the other hand, the actual evidence of vertigo is mostly due to the blockage of phlegm and turbidity, which leads to the upward obscuration of the clear orifices [9]. Therefore, this disease is the syndrome of deficiency in nature and excess in superficiality. Based on this, when formulating clinical treatment, we can start from the ideas of suppressing hyperactive liver for calmingendogenous wind, benefiting Qi and activating blood circulation, and disperse blood stasis and dredge collateral [15].

Guizhi Gegen decoction is composed of Ge Gen, Tian Ma, Gui Zhi, Bai Shao, Qiang Wu, Chuan Xiong, Sheng Jiang, Silique, and *Glycyrrhiza glabra*, which has the effect of relieving superficies, dispersing superficial exopathogens, and harmonizing yingfen and weifen [16]. *Pueraria mirifica* is one of the highest dose ingredients in this remedy, which has the effect of expelling pathogenic factors from muscles for clearing heat, relieving clinical symptoms such as exterior syndrome fever, and stiff nape and back [17]. The Tianma is sweet in taste and neutral-natured, which can stop endogenous wind and alleviate pain. It is pointed out in the Materia Medica Huiyan that tianma is used for head wind, headache, dizziness, and vertigo. Gui Zhi has the effect of dispelling cold to relieving pain and assisting yang and transform qi, so the combination with Tian Ma can enhance the efficacy of both. In addition, Bai Shao can nourish liver, alleviate pain, and stabilize liver yang. Chuan Xiong can regulate qi, which can treat wind-cold headache and dizziness. Ginger can dispel the exterior cold. Stiff silkworm can breathe wind and stop spasms, dissolve phlegm, and disperse knots. Licorice can reconcile various drugs [17].

Also, the modern pharmacological study on the pharmacology of Gui Zhi Ge Gen decoction shows that the effective component of *Pueraria* root was Radix puerariae total flavonoids, which can dilate vascular smooth muscle, reduce peripheral resistance, and increase local blood flow [18]. Also, Gui Zhi has the effect of promoting tissue metabolism and expanding blood vessels, and Gui Zhi, Licorice, and Bai Shao have both anti-inflammatory and analgesic effects. Therefore, Gui Zhi Ge Gen decoction can nourish cervical intervertebral disc cells while being anti-inflammatory and analgesic, so as to improve the symptoms and delay the degeneration of cervical intervertebral disc.

Due to the limitation of poor overall efficacy of single medication, the combination of electroacupuncture and medication is accepted by most clinicians in the treatment of cervical vertigo [19]. In this study, we investigated the clinical efficacy of electroacupuncture combined with Gui Zhi Ge Gen Tang on the basis of conventional treatment in Western medicine. The results showed that the effective rate of the study group was higher than that of the control group, and the ESCV score after treatment was higher than those before treatment and control group (*P* < 0.05). Electroacupuncture is a method of treating diseases by combining both needle and electrical stimulation by passing a trace current close to human bioelectricity through the needle tool after acupuncture into the acupuncture point to obtain qi [20]. In terms of acupuncture points, this study selected the cervical 4–7 jiaoji points as the main acupuncture points according to the clinical characteristics of cervical vertigo and took Tianzhu, bilateral Fengchi, Houxi, and Liji as the secondary acupuncture points with significant effects [21]. On the one hand, the pinched spine points are closely related to the nerve segments, and acupuncture of the pinched spine points can affect both the posterior branch of the spinal nerve and its anterior branch. Electroacupuncture stimulation can cause needle sensory conduction, which can alleviate the compression of the vertebral artery and cervical sympathetic nerve to a greater extent and relieve the current situation of obstructed blood flow in the vertebrobasilar artery. On the other hand, electroacupuncture treatment can improve the microcirculatory status, regulate capillary permeability, and increase tissue oxygenation and blood flow operation [22]. Therefore, electroacupuncture treatment can significantly reduce the symptoms of vertigo.

Insufficient vertebrobasilar blood supply, resulting in slow blood flow and high blood viscosity, is a key factor in the cause of vertigo [23]. The LVA, RVA, and VB can reflect the blood flow in the vertebrobasilar artery, while high cut whole blood viscosity, low cut whole blood viscosity, and plasma viscosity are commonly used indexes to reflect blood fluidity and viscosity [24]. The results of this study showed that, after treatment, LVA, RVA, and VB were higher in the study group than in the control group, and whole blood viscosity high cut, whole blood viscosity low cut, and plasma viscosity were lower than in the control group (*P* < 0.05). This indicates that electroacupuncture combined with Gui Zhi Ge Gen Tang can effectively improve the blood supply rate and blood viscosity of the vertebrobasilar artery. Quality of life is also an important index for evaluating clinical efficacy. The results of our study showed that the quality of life in the study group was significantly improved after treatment compared with before treatment (*P* < 0.05), but the scores of various indexes of quality of life in the control group after treatment were not statistically significant compared with that before treatment (*P* > 0.05). This result suggests that electroacupuncture combined with Gui Zhi Ge Gen Tang has a significant effect on improving clinical symptoms and quality of life of patients with cervical vertigo. Also, the results of adverse reaction investigation showed that there were no serious adverse reactions during and after treatment in both groups, which further confirmed the safety of electroacupuncture combined with Gui Zhi Ge Gen Tang in the treatment of cervical vertigo.

To sum up, electroacupuncture combined with Gui Zhi Ge Gen Tang can effectively increase the blood flow velocity of the vertebrobasilar artery in patients with cervical vertigo and improve their blood rheology and quality of life with precise efficacy and high safety. The shortcoming of this study was that the sample size was small. In the future studies, the sample size can be further expanded to study the pathogenesis of cervical vertigo in depth and provide scientific basis for clinical treatment.

## Figures and Tables

**Table 1:** Comparison of clinical efficacy between the two groups (*n* (%)).

Group	Recovery	Markedly effective	Effective	No effect	Total effective rate
Study group (*n* = 63)	29 (46.03)	19 (30.16)	12 (19.05)	3 (4.76)	95.24
Control group (*n* = 57）	25 (43.86)	13 (22.81)	10 (17.54)	9 (15.79)	84.21
*χ* ^2^	—	—	—	—	4.043
*P*	—	—	—	—	0.044

**Table 2:** Comparison of ESCV scores before and after treatment between the two groups ($\bar{x}\pm s$, score).

Group		Vertigo	Headache	Neck and shoulder pain	Daily life and work	Psychological and social adjustment
Study group (*n* = 63)	Before treatment	1.02 ± 0.35	1.23 ± 0.41	1.14 ± 0.36	1.19 ± 0.21	1.35 ± 0.49
	After treatment	2.43 ± 0.19^*∗*^	2.56 ± 0.24^*∗*^	2.36 ± 0.31^*∗*^	2.55 ± 0.16^*∗*^	2.36 ± 0.39^*∗*^

*t*		28.102	22.221	20.383	40.888	12.801

*P*		≤0.001	≤0.001	≤0.001	≤0.001	≤0.001

Control group (*n* = 57)	Before treatment	1.06 ± 0.29	1.21 ± 0.43	1.16 ± 0.40	1.13 ± 0.25	1.31 ± 0.52
	After treatment	1.89 ± 0.36	1.91 ± 0.46	1.85 ± 0.39	1.83 ± 0.32	1.93 ± 0.43

*t*		13.555	8.393	9.325	13.014	6.937

*P*		≤0.001	≤0.001	≤0.001	≤0.001	≤0.001

*Note*. Compared with the control group after treatment, ^*∗*^*P* < 0.05.

**Table 3:** Comparison of TCD before and after treatment between the two groups $\left(\bar{x}\pm s,\;\text{cm}/\text{s}\right)$.

Group		LVA	RVA	VB
Study group (*n* = 63)	Before treatment	22.39 ± 5.62	18.97 ± 4.46	25.71 ± 4.34
	After treatment	31.71 ± 4.95^*∗*^	28.11 ± 4.31^*∗*^	34.96 ± 5.61^*∗*^

*t*		9.878	11.697	10.351

*P*		≤0.001	≤0.001	≤0.001

Control group (*n* = 57)	Before treatment	23.44 ± 5.31	18.41 ± 4.63	25.94 ± 4.17
	After treatment	27.69 ± 5.32	24.31 ± 4.55	29.39 ± 5.15

*t*		4.269	6.862	3.931

*P*		≤0.001	≤0.001	≤0.001

*Note*. Compared with the control group after treatment, ^*∗*^*P* < 0.05.

**Table 4:** Comparison of blood rheological index levels before and after treatment between the two groups $\left(\bar{x}\pm s,\text{ mpa}\cdot \text{s}\right)$.

Group		Whole blood viscosity high cut	Whole blood viscosity low cut	Plasma viscosity levels
Study group (*n* = 63)	Before treatment	1.86 ± 0.65	15.92 ± 2.37	6.39 ± 1.13
	After treatment	1.13 ± 0.31^*∗*^	10.27 ± 1.19^*∗*^	4.21 ± 0.56^*∗*^

*t*		8.046	16.910	13.720

*P*		≤0.001	≤0.001	≤0.001

Control group (*n* = 57)	Before treatment	1.85 ± 0.67	15.87 ± 2.46	6.21 ± 1.15
	After treatment	1.57 ± 0.52	12.39 ± 2.15	5.28 ± 1.60

*t*		2.493	8.042	3.563

*P*		0.014	≤0.001	≤0.001

*Note*. Compared with the control group after treatment, ^*∗*^*P* < 0.05.

**Table 5:** Comparison of quality of life between the two groups before and after treatment ($\bar{x}\pm s$, score).

Group		PF	RF	RE	BP	GH	VT	SF	MH	HT
Study group (*n* = 63)	Before treatment	71.56 ± 5.95	78.31 ± 4.37	72.82 ± 5.83	76.41 ± 5.12	75.18 ± 6.37	73.69 ± 6.39	75.82 ± 4.69	73.85 ± 6.17	72.63 ± 5.28
	After treatment	85.39 ± 5.41^*∗*^	84.66 ± 6.38^*∗*^	84.41 ± 6.39^*∗*^	84.96 ± 7.60^*∗*^	86.39 ± 6.98^*∗*^	83.17 ± 7.39^*∗*^	86.49 ± 5.34^*∗*^	86.97 ± 5.37^*∗*^	82.39 ± 6.49^*∗*^

*t*		13.650	6.518	10.635	7.406	9.416	7.702	11.916	12.731	9.259

*P*		≤0.001	≤0.001	≤0.001	≤0.001	≤0.001	≤0.001	≤0.001	≤0.001	≤0.001

Control group (*n* = 57)	Before treatment	71.69 ± 5.73	78.62 ± 4.51	73.12 ± 5.41	76.86 ± 5.33	75.26 ± 6.54	73.97 ± 6.41	76.08 ± 4.52	73.09 ± 6.48	72.51 ± 5.43
	After treatment	79.31 ± 5.98	80.96 ± 5.71	76.33 ± 6.12	79.97 ± 6.58	80.36 ± 5.79	78.39 ± 5.41	80.39 ± 5.96	80.16 ± 5.33	76.39 ± 7.31

*t*		7.303	2.553	3.119	2.915	4.634	4.183	4.573	6.688	3.382

*P*		≤0.001	0.012	0.002	0.004	≤0.001	≤0.001	≤0.001	≤0.001	≤0.001

*Note*. Compared with the control group after treatment, ^*∗*^*P* < 0.05.

## Data Availability

The data supporting the results of this study are available on reasonable request to the corresponding author.
